# Radioimaging Presentation of a Primitive Neuroectodermal Tumor of the Lung in a 13-Year-Old Female: A Case Report

**DOI:** 10.7759/cureus.60820

**Published:** 2024-05-21

**Authors:** Alushika Jain, Shivali V Kashikar, Rajasbala Dhande, Pratapsingh Parihar, Amit Toshniwal

**Affiliations:** 1 Radiodiagnosis, Jawaharlal Nehru Medical College, Datta Meghe Institute of Higher Education and Research, Wardha, IND; 2 Respiratory Medicine, Jawaharlal Nehru Medical College, Datta Meghe Institute of Higher Education and Research, Wardha, IND

**Keywords:** pediatric pnets, pleural mass, neoadjuvant therapy, neuroectodermal tumors, pnets, small round cell tumors

## Abstract

Primitive neuroectodermal tumors (PNETs) are unprecedented threatening neoplasms beginning from primitive neuroectodermal cells. PNETs are reported as the predominant incidence observed in children and young adults with a high mortality rate. These neuroectodermal tumors are quite aggressive with a life expectancy of eight months on average. PNETs belong to the family of small round cell tumors majorly affecting bones and soft tissues in different body parts such as the brain, lungs, spine, and pelvic region. Computed tomography (CT) and magnetic resonance imaging (MRI) play a major role in giving the size, extent, and resectability of the tumors. A confirmed diagnosis is then made by histopathology and immunohistochemistry markers. This report depicts a case of PNET found within the right lung of a 13-year-old female, enumerating the clinical introduction, demonstrative handle, treatment modalities, and results. The case underscores the significance of precise conclusions and multidisciplinary approaches in pediatric PNET cases. Once the provisional diagnosis of pleuropulmonary blastoma or PNET was given on CT, a conformational histopathological examination was carried out. Histopathological analysis confirmed the final diagnosis of PNET, and the patient underwent neoadjuvant therapy as the tumor was non-resectable due to its massive size.

## Introduction

Primitive neuroectodermal tumors (PNETs) are aggressive malignancies emerging from primitive neuroectodermal cells, essentially watched within the central apprehensive framework but can moreover show in extracranial areas, such as the lung [1]. PNETs are reported to be identical to "Ewing's sarcomas" due to the same chromosomal translocation. Both these tumor types can be noted as the same tumor variants attributing similar clinical presentations with varying degrees of neuronal differentiation [1,2]. PNETs are neuroectodermal malignancies, often affecting the soft tissues and the bones. PNETs represent 4-17% of all juvenile soft tissue cancers and are reported as extremely malignant neoplasms frequently observed in bone and soft tissues [3]. PNETs are aggressive malignancies from small round cell tumors, which can be differentiated based on immunohistochemistry [1]. Common clinical symptoms depend on the location of PNETs which include seizures, memory issues, headaches, imbalance issues, numbness, and weakness [4]. Common clinical symptoms depending on this particular PNET of the lung were observed as breathlessness, right-sided chest pain, and dry cough. PNETs are most commonly observed in children and adolescents, with most cases reported in young adults under 30 years of age [5]. A five-year survival rate of the PNET-affected individuals is reported only between 5 and 10% [1]. Hence, in this case, the PNET being so large in size, surgery was not recommended, and neoadjuvant chemotherapy was given. PNETs are aggressive and have a high risk of metastasis and reoccurrence [1,3-5]. A multimodal therapeutic approach is required for Ewing's sarcoma family. Generally, surgical resection is recommended, though a multidisciplinary approach by neoadjuvant chemotherapy is recommended to improve the prognosis and to prevent recurrence [5]. A very low life expectancy is expected with PNETs with an average duration of 3-9 months in a few cases [5,6]. This is the case of a 13-year-old female with PNET in the right lung, highlighting the need for inciting determination and comprehensive treatment.

## Case presentation

A 13-year-old female visited the outpatient department, with a persistent history of intermittent fever, cold, cough with expectoration, dyspnea, and dynamic right-sided chest pain in the last three months. She was otherwise healthy or asymptomatic three months ago. Physical examination revealed diminished breath sounds over the right lung base. An initial diagnostic workup X-ray was done, which showed a white-out lung and total right hemithorax opacification. Radiological screening by an X-ray revealed a pulmonary mass spreading in the lower and medium parts of the thorax and blunting of the cardiophrenic angle and costophrenic angle on the right side with left-sided mediastinal shift, which was initially thought to be a massive right-sided pleural effusion (Figure 1).

**Figure 1:** A close view of the X-ray image of the patient showing a large rounded opacity almost involving the whole of the right lung with a convex margin upward, probably right lung mass

Ultrasonography (USG) was done which showed bilateral pleural effusion, right>left, and hence, the intercoastal tube insertion was done on the right side, and about 250 CC fluid was drained. The child was given empirical treatment (azithromycin and amoxicillin) for two weeks with no positive outcome. The patient was subjected to a blood workup, chest X-ray, computed tomography (CT), and magnetic resonance imaging (MRI). Blood investigations showed a rise in total leucocyte count, and sputum culture showed the presence of pus cells, which raised a suspicion towards differentiating an infective etiology from malignancy. A high-resolution computed tomography (HRCT) of the thorax was then advised and done, revealing an unexpected outcome: a noteworthy mass within the right lung base reaching up to the apex.

Diagnostic workup

HRCT of the thorax revealed a well-defined pleural-based (broad-based towards pleura) heterogeneous mass lesion with intense internal septation and hypodense areas noted in the right hemithorax measuring 9.1 × 8.5 × 9 centimeters. The lesion extends to the posterior and middle mediastinum, causing a mass effect in the form of mild displacement of great vessels, viz., arch of aorta, descending aorta, and cardia towards the left side. The lesion is seen abutting the descending aorta (180 degrees) and right atrium, along with the compression of the right pulmonary artery. The right main bronchus is seen obliterated. Bilateral axillary lymphadenopathy is also seen. Bilateral pleural effusion was noted (right>left) with an intercoastal drainage tube within the right pleural cavity in the region of the posterobasal segment of the right lower lobe (Figure 2, Figure 3). 

**Figure 2:** CT axial section of the lung window showing right lung mass CT: computed tomography

**Figure 3:** CT axial section of the mediastinal window showing large right-sided mass causing a mediastinal shift to the left CT: computed tomography

Dorsal spine MRI showed evidence of altered signal intensity solid cystic lesion in the right hemithorax with broad-based pleura and appearing hyperintense on T2-weighted imaging (T2WI)/T1-weighted imaging (T1WI)/short tau inversion recovery (STIR) and collapse of basal segments of the right lower lobe and similar findings to that of HRCT of the thorax. D6 vertebra showed a lytic and sclerotic lesion, which is most likely to be metastasis (Figure 4).

**Figure 4:** MRI sagittal section of the whole spine showing normal spinal canal diameter and a lytic lesion at the D6 vertebra most likely to be metastasis MRI: magnetic resonance imaging

The MRI also showed that there were normal spinal canal diameter and no evidence of spinal cord compression or myelopathy (Figure 5, Figure 6).

**Figure 5:** MRI sagittal section of the right hemithorax (A) T2WI, (B) T1WI, and (C and D) T2WI STIR showing altered signal intensity solid cystic mass with its extent MRI: magnetic resonance imaging; T2WI: T2-weighted imaging; T1WI: T1-weighted imaging; STIR: short tau inversion recovery

**Figure 6:** MRI of the right hemithorax (A and B) T2WI/STIR (coronal), (C) T2WI (axial), and (D) T1WI (axial) heterogeneously hyperintense solid cystic lesion in the right hemithorax with the collapse of segments of the right lower lobe with extension into the posterior and middle mediastinum MRI: magnetic resonance imaging; T2WI: T2-weighted imaging; T1WI: T1-weighted imaging; STIR: short tau inversion recovery

A squash cytology of the tissue collected by needle aspiration of the pleura-pulmonary mass was done. The smears showed multiple small groups and sheets of small cells placed cohesively along with cellular crowding in the center of the group. These cells were circular, blue cells with insufficient cytoplasm and hyperchromatic cores. The nuclei showed mild pleomorphism and granular yet condensed chromatin, which is irregular. The background showed hemorrhagic material and few nuclear debris. Immunohistochemical examination illustrated for CD99, NKX2.2, EMA, and neuron-specific enolase (NSE), reliable with PNETs. Molecular analysis affirmed EWSR1 gene rearrangement, affirming the diagnosis (Figure 7).

**Figure 7:** Immunohistological staining of the pleura-pulmonary mass (A) Hematoxylin and eosin stain showing circular, blue cells with insufficient cytoplasm and hyperchromatic cores. (B) Positively stained for CD99. (C) Positively stained for NKX2.2

Treatment and outcome

PNETs are very aggressive tumors, and usually, surgery is recommended as they have a high chance of recurrence. A multidisciplinary approach is required for Ewing's sarcoma family. The patient was managed by neoadjuvant therapy, as surgery was not possible, due to the massive size of the tumor and also the suspicion of metastasis in the vertebral column. She underwent a combination of chemotherapy and radiotherapy. Surgical resection was then recommended for further treatment as the tumor had shrunk. Hence, the patient was advised surgical excision on the basis of the improvement noted after the treatment regime by neoadjuvant therapy which was vincristine (2 mg/m^2^) on day 1, doxorubicin (37.5 mg/m^2^) on days 1 and 2, cyclophosphamide (1200 mg/m^2^) on day 1 with mesna, and filgrastim (5 microgram/kg/day) on day 3. She then underwent a successful right lung pneumonectomy with no post-operative complications. The patient had a one-month hospital stay and showed good improvement. Further, the patient was suggested a follow-up with re-evaluations for PNET status until two years post-operative so as to rule out recurrence.

## Discussion

PNETs happening in extracranial organs, such as the lung, pelvis, retroperitoneum, and neck, are uncommon and reported to progress rapidly with high mortality and recurrence rates [3]. Generally, PNETs on imaging have no clear boundary, are very heterogeneous, and invade surrounding tissues as they progress, making it challenging to report and surgically resect [5]. This case report acclimates to proficient measures and gives a comprehensive diagram of PNET within the right lung of a 13-year-old female child. PNETs associated with the lungs have been reported to have no correlation with smoking in adults. These tumors have also been reported with a very poor prognosis and a common metastatic presentation noted when the disease is first diagnosed as observed in this case [7]. PNETs on the basis of radiological imaging modalities such as X-ray, MRI, and CT can be observed as heterogeneous masses of intrapulmonary nature which are found to be commonly invading the adjacent tissues, without any distinct feature as compared to other lung tumors [8]. PNETs when observed in the lungs are recommended additional tests such as a positron emission tomography (PET) scan of the surrounding tissues and bones and a biopsy of the bone marrow, to rule out the metastasis. Immunohistochemical tests, histopathological examinations, and molecular analysis can be helpful in the confirmation of lung PNETs attributed to the absence of distinctive radiological features and poor prognostic outcomes [3,7,8]. Few research have shown that molecular markers, such as MIC2 and EWS-FLI1, can be used for the differentiation of PNETs of the central nervous system and those arising out of the autonomic nervous system, which can be helpful in the decision of the course of disease management [7,9]. A multidisciplinary approach, including chemotherapy, surgery, and radiation treatment, is basic for better outcomes [10].

## Conclusions

PNET within the lung poses critical challenges, requiring a multidisciplinary approach for a good outcome. Also, it poses a challenge for the diagnosis carried out only by imaging modalities. Histopathological examination and immunohistochemistry are recommended for a confirmatory final diagnosis. Surgery and chemotherapy are the ideal treatments, while large lesions are treated with neoadjuvant chemotherapy followed by surgery though good outcomes are expected. Convenient determination and multidisciplinary treatment approach are basic for upgrading results in pediatric patients with PNET. However, there are instances showing large PNET masses being treated surgically with success after chemotherapy. Long-term surveillance is fundamental for checking potential recurrence and treatment-related complications. Collaboration among healthcare providers is imperative to conveying comprehensive care to these patients.
